# Chinese Public Perception of Climate Change on Social Media: An Investigation Based on Data Mining and Text Analysis

**DOI:** 10.1155/2022/6294436

**Published:** 2022-08-24

**Authors:** Li Zeng

**Affiliations:** Department of Journalism and Communication, South China Normal University, Guangzhou, China

## Abstract

Climate change is a serious threat to humankind. As broad public participation is required in climate change mitigation efforts, it is critical to understand how the public talk about climate change on social media. This study sets out to increase the understanding of Chinese public awareness of climate change, as well as explore the potential and limitations of social media for public engagement on climate change issues. It examines the Chinese public's discussion about climate change on social media Weibo during the last six years through data mining and text analysis. The analyses include volume analysis, keyword extraction, topic modeling, and sentiment analysis. The results indicate three main aspects of public awareness and concern regarding climate change. First, public awareness of climate change is growing in China. Second, the sentiment analysis shows that the general sentiment toward climate change is becoming more positive over time. Third, based on keyword extraction and topic modeling, the discussion on climate change shows a top-down perspective, an optimistic economic perspective, and a preference for celebrity content. The study provides a comprehensive picture of Chinese social media users' views on climate change issues, based on large-scale research data. It contributes to a better understanding of what Chinese people think about climate change on social media generally. These findings may provide government and environmental organizations with valuable insights for better climate change campaigns on social media.

## 1. Introduction

Climate change is a serious threat to humankind. It refers to the change in climate patterns due to greenhouse gas emissions [1]. Recent research indicates that it has serious effects on human society, including more frequent extreme temperatures, flooding, threats to food security, and reduced economic growth [2–4]. Furthermore, climate change could have a negative impact on the individual's physical and mental health [5, 6] (Costello et al., 2009; Hayes et al., 2018).

The COVID-19 pandemic has made a complex impact on climate change. On the one hand, the pandemic limits economic activity and reduces energy consumption and greenhouse gas emissions [7, 8] (Wang & Su, 2020; Wang, Li & Jiang, 2021). On the other hand, the epidemic has the potential to reduce the concern for climate change, resulting in a neglect of climate change issues [9] (Phillips, Caldas & Cleetus, 2020).

The scientific community has widely accepted that climate change occurs because of human activity [10]. Therefore, broad public participation is required in climate change mitigation efforts. Public participation in climate change discussions is considered to resolve differences and promote action [11]. Social media, with its decentralized and participatory nature [12], is becoming a significant platform for information exchange, opinion formation, and public affairs engagement [13]. Therefore, it is critical to understand how the public talk about climate change on social media.

A large and growing body of literature has investigated the discussion of climate change on social media. These studies mainly fall into three categories:

1. the public's overall attitude towards climate change, including its overall trend of the change, and whether climate change is perceived to be true [10];
2. public discussion on a particular climate change event, such as responding to a particular extreme weather event [14, 15];
3. how Twitter motivates people to act on climate change [16, 17].

Most studies in this field have only focused on social media in the USA and Europe, with few studies from developing countries [18]. However, China, the world's largest emitter of greenhouse gases, is a global climate governance power to be reckoned with [19]. Along with the United States, China is increasingly becoming a critical leading force in global climate change. In the context of the COVID-19 epidemic especially, the recovery of the Chinese economy after the epidemic has a spillover effect on other countries' energy consumption [20] (Wang & Zhang, 2021). In such a context, it is essential to study the attitudes of the Chinese public toward climate change.

With 573 million monthly active users, Weibo is one of China's largest social media platforms [21]. It has become an essential platform for investigating people's attitudes towards public events [22, 23].

While some research has been carried out on climate change in Chinese social media, an overall view has not been established. These studies mainly focus on a particular climate change event, such as discussions on Weibo about the Paris summit and the Chinese government's climate change report [24, 25]. They provide insight into the Chinese public's perceptions of climate change but lack a comprehensive picture. It is still unknown how Chinese people discuss climate change in general. What exactly are their attitudes toward climate change? Additionally, because sentiment is critical for information dissemination and social mobilization, it is vital to measure the collective sentiment [26, 27].

Therefore, the main aim of this study is to investigate the discussion of climate change on Chinese social media (Weibo). By crawling all the data on climate change for a long time (six years), we tried to answer the following questions. (1) How does the level of concern about climate change on Weibo change among Chinese people? (2) What are the primary topics of discussion on Weibo regarding climate change? (3) How do Chinese people feel about climate change when they discuss it on Weibo?

This study contributes to the existing literature in two ways. First, it provides a useful research framework for studying environmental issues on social media. Computer-assisted text mining techniques and methods are used in the paper, which reduces the subjectivity associated with questionnaires and interviews. Second, the study provides a six-year longitudinal analysis of social media data, which provides a more comprehensive picture of public perceptions of climate change.

## 2. Materials and Methods

As shown in Figure 1, the study has three main stages: data collection, data preparation, and data analysis, and the specific steps are as follows.

1. *Data Collection.* This study used python to collect data from Sina Weibo (https://www.weibo.com) with the post containing “气候变化” (climate change). The collecting period was set from 12 December, 2015, to 12 December, 2021, six years after the Paris Climate Summit. 388193 posts were collected.
2. *Data Cleaning.* After data cleaning, duplicates and irrelevant data were deleted. A total of 346921 posts were gathered.
3. *Data Preprocessing.* In this paper, we employed Jieba module for Chinese word segmentation. Then, we removed the stop words from the segmentation results.
4. *Volume Analysis.* By describing and analyzing the volume of posts generated from Weibo over time, we may better understand its trend and characteristics.
5. *Keyword Extraction.* We employed keyword extraction methods with different term weights using TF-IDF and TextRank.
6. Topic Modeling. We trained an LDA model on the data corpus using Python's Gensim library. We chose 16 as the topic number for our final topic model, based on perplexity curves.
7. *Sentiment Analysis.* This paper called SnowNLP to do the sentiment analysis of the Weibo posts. The sentiment value of each post is automatically calculated, and outputting results are between 0 and 1. The closer it gets to 1, the more positive the emotion is, and the closer it gets to 0, the more negative it is.

## 3. Results

After completing the previously mentioned steps, the results were as follows.

### 3.1. Volume Analysis Results

In this section, we analysed the variation in the number of posts (volume) discussing climate change over time, as shown in Figure 2.

Through the analysis of the volume of posts, we could identify the various levels of awareness and discussion about climate change-related topics. Figure 2 presents a clear trend of an increase in the overall volume of these posts over time.

There are different stages of this upward trend. There are a few posts before March 2018, and then, it rises. By examining the content of March 2018 posts, there might be two probable explanations for the change. One is that the Earth Hour was held on March. And from that year, WWF began to invite some celebrities and influencers who were popular among Chinese youth. So, many fans' posts mentioned the Earth Hour and climate change. The other is that China established the Ministry of Ecology and Environment in March 2018, indicating that China will maintain its unprecedented commitment to and investment in climate change mitigation in the future [28]. It is worth noting that there is a decline in discussion between February and June 2020, possibly because of the impact of the COVID-19 epidemic.

Then, we counted the number of posts for each month, and the figure is as follows. It shows that there has been an increase in March, November, and December. This is partly attributed to climate change events such as the Earth Hour and the Conference of the Parties (COP). The former is held in March, while the latter is usually held in November or December. Another reason might be that the most critical environmental issue for the Chinese public is haze, which usually occurs during the fall and winter. Many Chinese people considered climate change and haze as the same thing.

### 3.2. Keyword Analysis

The keyword extraction is a commonly used text mining task that involves identifying a set of terms that best describe the text. In this section, we will perform keyword extraction with TextRank and TF-IDF.

Table 1 lists the top 20 keywords after both algorithms were used. As the table shows, 80% of the words extracted by the two methods are consistent, showing that the extraction method is reliable.

These keywords reflect a top-down perspective. The words China, the United States, global, Earth, national, world, cooperation, human, international, and conference convey an image of humankind cooperating to combat climate change through the political cooperation.

In particular, the keywords bring a national perspective. China is the top two keyword in both algorithms, while the United States is also mentioned in both algorithms. Interestingly, both China and the United States are ranked higher than the United Nations. It might suggest that Chinese public opinion views climate change as a bilateral issue between China and the US. And their cooperation sometimes goes beyond the UN framework.

It is worth noting that the star's name, Zheng Shuang, occurs in the keywords. Zheng Shuang is a well-known Chinese actress with over 10 million Weibo followers. Her name appears in several posts since she has taken part in various UN climate change campaigns [29]. It is partly due to the TF-IDF's algorithm, which prioritizes terms that are not prevalent in the context. It does, however, indicate a significant role for celebrities in impacting Chinese public opinion about climate change.

### 3.3. Topic Modeling

The topic modeling process was carried out on the text field of climate change-related posts to understand the main themes of the discussions.

The Latent Dirichlet Allocation method is commonly used for document modeling, text classification, and collaborative filtering.  Table 2 shows that 16 topics were identified with the top relevant keywords, and topic names were assigned manually to each topic.

Next, the topic names were ranked in descending order based on the number of posts relevant to the topic, as shown in Figure 3.

We obtained the following findings through the distribution of topics.

1. The economy perspective, which includes keywords like projects, firms, and investment, is the most frequently discussed topic on Weibo.
2. There have been numerous conversations about gas emissions and energy saving, which indicates that climate change and gas emissions are regarded quite related.
3. There are also many discussions on Sino-US cooperation. In the context of climate change, the most frequently discussed international cooperation is China and the United States. The result shows the Chinese public's view of climate change as a global issue that cannot be resolved by the efforts of a single country. Likewise, it reflects the Chinese public's perception of Sino-US cooperation as being superior to any other cooperation.
4. Finally, there is little discussion on the food crisis, probably because the Chinese public rarely experience it; hence, they do not perceive it strongly enough.

Furthermore, the paper examines how the proportions of the topics have changed over time. See Figure 4.

According to the changes in the graph, some topics have remained important, while others have changed over time. The former includes the economic perspective, which has always been given a greater weight, showing that this is the primary concern. The latter covers topics such as everyday actions and energy savings and emission reduction. Everyday actions declined with time, while energy savings and emission reduction was less crucial in the beginning but became more critical with time. To some extent, this reflects the shift in the focus of climate change from a personal to an industrial issue, that is, the recognition that manufacturing produces more greenhouse gases than the individual's daily use [30].

Moreover, as seen in Figure 5, these topics could be classified into three broad groups.

1. *Phenomenon Group.* It describes the phenomenon of climate change and includes topics 8 (research data) and 11 (gas emissions). They focus on the greenhouse gas emissions as causes of climate change. They also show the research that reveals the status of global climate change.
2. *Consequences Group.* This section covers topics 3 (human health), 5 (influence), 6 (global warming), 7 (food crisis), and 14 (air pollution). They discuss the consequences of climate change, which include global warming, food crisis, atmospheric problems, and harmful effects on human health.
3. *Solutions Group.* This contains topics 1 (China's response), 2 (Sino-US relations), 4 (economic perspectives), 9 (United Nations framework), 10 (environmental campaign), 12 (biological conservation), 13 (youth action), 15 (everyday actions), and 16 (energy saving and emission reduction). They focus on measures to address climate change. Political and economic measures are included, as well as environmental promotion and the mobilization of young people to make climate change a daily practice.

When the distribution of the number of topic group is viewed further, solutions group account for most of the proportions.

### 3.4. Sentiment Analysis

We performed sentiment analysis to gauge how the public feels about climate change. In this study, through SnowNLP, each Weibo content is assigned a sentiment value, ranging from 0 to 1. The closer it is to 0, the more negative the sentiment is, and the closer it is to 1, the more positive the sentiment is. At the same time, 0.5 is used as the dividing point between positive and negative. If it is less than 0.5, it will be marked as positive sentiment, and if it is greater than or equal to 0.5, it will be marked as negative sentiment.

Table 3 shows that negative content describes climate change-related disasters, and positive content tend to emphasise efforts to combat it.

It can be observed from Figure 6 that the number of positive posts exceed that of the negative ones during the research time. And there is more extreme content in both positive content and negative ones.

Figure 7 shows the change of sentiment over time. We can see from the graph that the number of positive and negative is increasing with time and that the content of positive emotions is increasing at a faster rate than the content of negative ones.

Figure 8 shows how sentiment analysis has performed throughout various months. Generally, negative emotions are higher in the fall and winter. This is in line with prior research that people are more likely to feel happy when the weather is warmer [31]. However, the only exception is December, when the mood is more positive than other fall and winter mouths. One explanation is that climate conferences are often held in December, resulting in a flurry of positive posts on constructive efforts.

The average of the sentiment value for different topics was shown in Figure 9.

The sentiment value is more positive when it comes to the topic on solutions such as energy conservation, youth action, and Sino-US relations but is somewhat negative when it comes to environmental campaign, research data, and gas emissions. Interestingly, topic 10 (environmental campaign) is relatively negative. This might be because this topic tends to highlight the cost of being environmentally unfriendly to raise public awareness of climate change issues.

## 4. Discussion

Based on the data analysis presented in this paper, we have identified the following characteristics of climate change discussions on Weibo.

One noteworthy finding is climate change viewed from a top-down perspective. The top-down perspective refers to the view of climate change from a national rather than an individual or local perspective. It is demonstrated in the keyword extraction process, where words such as China, world, global, and international are highly ranked. Additionally, the topic modeling shows that the amount of content related to international cooperation and national response measures is much greater than individual actions. This is contrary to the findings of Dahal et al. (2019), who determined that discussions on Twitter were less likely to involve top-down advocacy for climate change [26].

The top-down perspective may be attributed to China's own political ecology and mobilization approach [32–34]. Yang (2021) argues that the discussion of climate change in China lacks bottom-up information flow [25]. Pan (2020), in his discourse analysis of Chinese journalists, suggests they view climate change as a policy issue, emphasizing the central role of the Chinese government [35].

Furthermore, this implies that the Chinese people themselves do not regard climate change as a tangentially relevant issue. Liu (2017) notes that Chinese people consider climate change to be a global threat unrelated to China's own conditions [24]. In fact, the Chinese are most concerned with haze when it comes to environmental concerns [36, 37]. When asked “what comes to mind when you hear about climate change,” about 6.3% of people think of haze, ranking second among all words [38].

As a result of this top-down perspective, climate change policies in China may not encounter the same fierce opposition as they do in the United States [13]. However, the public opinion on Weibo suggests that climate change is not perceived as a personal concern. It is the result of government initiative with little bottom-up participation from the people. Further, it raises the concern whether Weibo can actually encourage public action on climate change.

Second, a significant proportion of the Chinese public's discussion of climate change on Weibo revolves around economic aspects and maintains an optimistic attitude.

As shown in the topic modeling, the economy is the most frequently discussed topic on Weibo. It is consistent with the view of Bill Gates, who regards climate change as an economic issue and emphasizes the importance of addressing it both economically and technologically [39].

Additionally, the Chinese populace perceives climate change as a potential economic opportunity. While China is facing many challenges because of climate change, policy makers and researchers see it as an opportunity for the country's economic transformation. As for traditional energy, China is an importer, while for new energy, China has the world's largest installed capacity of wind power, solar power, and hydropower and is a leading force in this field [40].

Taking these findings into account, we might gain a better understanding of the Chinese complex view on climate change, regarding it as both a threat and an opportunity.

Finally, what is surprising is that celebrities and stars play a significant role in the climate change discussion. According to the keyword analysis, the names of celebrities appear at the top of the list. Additionally, WWF's Earth Hour in China would not have attracted such attention without the involvement of celebrities, especially those with huge followings.

This result is partly due to the entertainment-oriented nature of Weibo itself [41], but it is also a worldwide phenomenon [42]. The celebrity effect has a complex effect. On the one hand, it raises public awareness of climate change. On the other hand, there are concerns that celebrity involvement in climate change “renders behavior change insignificant and condones continued consumerism [43, 44].”

An analysis of celebrities' relevant Weibo posts reveals that they mainly repeat slogans rather than providing specific guidelines for converting slogans into practical actions. Additionally, most of the comments made by the celebrities' fans on the related posts admire celebrities for their social responsibility, while ignoring the issue of climate change itself.

## 5. Conclusions

Climate change poses a serious threat to humankind. Broad public participation is necessary for climate change mitigation efforts, so it is important to understand how the public uses social media to discuss climate change.

The purpose of this study is to gain a deeper understanding of Chinese public awareness of climate change, as well as examining the complex role that social media play in promoting public engagement with climate change issues. We employed volume analysis to measure the level of concern about climate change, keywords, and latent distribution analysis (LDA) to decipher the topic of climate change and sentiment analysis to understand public opinion about climate change issues.

The main conclusions of this study are as follows.

1. Chinese people's concern about climate change is gradually increasing on social media, although it fluctuates based on special events. Some government policies and campaigns can increase social media discussions. However, major public health issues, like the COVID-19 pandemic, can divert attention and reduce discussions in the short term.
2. Attitudes towards climate change in China are positive on social media, and it correlates with the topics discussed and the posting date. The sentiment analysis shows that the general sentiment toward climate change is becoming more positive over time. It shows that negative content describes climate change-related disasters, and positive content tends to emphasise the efforts to combat it. Besides, negative emotions are higher in the fall and winter.
3. The content of the discussion shows a top-down perspective, an optimistic economic perspective, and a preference for celebrity content. First, many climate-relating posts on Weibo share the view of climate change from a national rather than an individual or local perspective. The public opinion on Weibo suggests that climate change is not perceived as a personal concern. However, concerns have been raised about its ability to really mobilize the public because of its lack of meaningful discussion and attention from the bottom-up. Second, despite climate change's challenges, many Chinese see it as an opportunity for China's economic transformation. Third, celebrities and stars play a significant role in climate change discussion.

According to this study, social media platforms provide a valuable tool for environmental communication, so the government and environmental organizations could take advantage of them. Several specific suggestions can be summarized based on our empirical results: First, a bottom-up perspective on climate change should be emphasized on social media, which stresses that climate change is a public event relevant to everyone. Personalized narratives can be added to change the focus from “climate change is important” to “what can I do to combat climate change?” Second, it is also important to take advantage of the celebrity effect. Celebrity narratives can enhance the appeal of environmental communication, particularly among young people.

The study has some limitations.

  First, users on Weibo are relatively young and therefore do not fully represent China's public opinion [45]. Then, this study treats the Chinese public as a homogeneous group without considering its internal differences, such as geography and gender.
  This research has thrown up many questions in need of further investigation. To understand a broader range of Chinese people's attitudes toward climate change, further research should be conducted involving a broader range of platforms, such as WeChat and TikTok. Further studies are needed to examine the influence of factors such as geography and gender.
  Further, this study reveals the positive attitudes of the Chinese towards climate change. However, the question whether such attitudes can be translated into positive actions remains to be answered. This would be a fruitful area for further work.

## Figures and Tables

**Figure 1:** Methodology.

**Figure 2:** Volume of posts across time.

**Figure 3:** Number of topics distributed.

**Figure 4:** Proportional change of each topic. The figure shows the percentage of a particular topic that appears each month. Based on this figure, we can see how the proportion of different topics has changed over time.

**Figure 5:** Distribution of the number of topic group.

**Figure 6:** The distribution of the number of each sentiment value.

**Figure 7:** Number of positive and negative posts over time.

**Figure 8:** Sentiment analysis of different months.

**Figure 9:** Average of sentiment value for different topics.

**Table 1:** Top20 keywords with TextRank and TF-IDF.

Rank	Text Rank	TF-IDF
1	Climate change	China
2	China	Global
3	Global	Zheng Shuang
4	Development	Address
5	Address	Earth
6	Climate	Climate
7	U.S.	Development
8	Earth	Action
9	Nation	Green
10	World	World
11	Problem	U.S.
12	Green	Protect
13	Cooperate	United Nations
14	Influence	Influence
15	Research	Problem
16	Environment	Humanity
17	Humanity	Environment
18	Action	Together
19	Protect	Cooperate
20	International	Conference

**Table 2:** Summary of LDA modeling result.

Topic	Topic name	Keywords
1	China's response	Development, response, China, green, build.
2	Sino-US cooperation	China, U.S.A, world, cooperation, country.
3	Human health	Attention, human body, disease, patient, treatment.
4	Economic perspective	Project, company, investment, market, enterprise.
5	Influence	Influence, human being, Earth, environment, problem.
6	Global warming	Global, air temperature, rise, global warming, sea level.
7	Food crisis	Population, food, research, yield, hunger.
8	Research data	Research, science, satellite, glacier, data.
9	United Nations framework	Paris, agreement, assembly, the United Nations, response.
10	Environmental campaign	Activity, environment protection, topic, campaign, follow.
11	Gas emission	Energy, carbon emission, greenhouse gas, carbon dioxide, clean.
12	Biological conservation	Global, ocean, protect, Antarctica, biology.
13	Youth action	Together, green, action, youth, ambassador.
14	Air pollution	Haze, emergency management, heating, pollute, pm 2.5.
15	Everyday actions	People, everyday simple, achieve, attention.
16	Energy saving and emission reduction	Energy saving, emission reduction, bluesky, green, low-carbon.

**Table 3:** Examples of content and sentiment value.

Content	Value	Positive/Negative
“The State Council Information Office held a press conference this morning (27) to release the 2019 Annual Report on China's Policies and Actions to Address Climate Change. After preliminary accounting, China's carbon dioxide emissions per unit of gross domestic product (GDP) fell by 4.0% in 2018, a cumulative decrease of 45.8% from 2005, equivalent to an emission reduction of 5.26 billion tons of carbon dioxide, and the proportion of non-fossil energy in total energy consumption reached 14.3%, basically reversing the rapid growth of carbon dioxide emissions.”	0.818	Positive
“As humans, we all want to build a beautiful house. Humanity is a community of destiny, both profitable and damaging faced with ecological and environmental issues, and no country can accomplish it alone. Only via collaboration will we be able to effectively address global environmental concerns such as climate change, marine pollution, and biological conservation, as well as to accomplish the United Nations' Sustainable Development Goals for 2030. Only by walking alongside one another can we ensure that the concept of green development takes root in people's hearts and minds and that the path toward a global ecological civilisation is steady and far-reaching.”	0.9853	Positive
“Pingxiang heavy rain I would like to say that the next-door Liling is the same. July days, there is still 22 degrees. Global climate change is getting more and more serious. When I went out today to find flooded areas after two days of heavy rain.”	0.0533	Negative
“[Polar bear wanders hundreds of miles to Russian city to find food in the garbage] On June 18, a hungry polar bear appeared in the suburbs of the northern industrial city of Norilsk, Russia. It is thin, bony, and slow-moving, rummaging through garbage dumps, searching for food. Because of its poor health condition, it is not suitable to be returned directly to its natural habitat. In recent years, the natural habitat of polar bears has been severely damaged by climate change and melting sea ice.”	0.0034	Negative

## Data Availability

All the data are available by contacting the author.
